# Research on the Innovative Development of Network Literature and Art under the Background of Mobile Digitalization

**DOI:** 10.1155/2022/8576522

**Published:** 2022-09-17

**Authors:** Bingyan Tang

**Affiliations:** School of Literature and Media, Xinyu College, Xinyu 338004, Jiangxi, China

## Abstract

The development of the times, the advancement of technology, and the innovation of the Internet have formed the soil for the growth of network literature and art. At present, there are still problems in the network literature and art, such as mixed fish and dragons, low quality, emphasis on entertainment, and weak responsibility, but its development is expected. Network literature and art is the product of the combination of literature and art and the development of science and technology. Meanwhile, network literature and art are an important part of social and economic development. It needs to seize the new opportunities of mobile digital technology to empower the creation, production, and dissemination of online literary and artistic works. Control the quality of online literature and art, guide its positive dissemination, and make it contribute to the prosperity of the entire Chinese literature and art.

## 1. Introduction

The development and prosperity of network literature and art is one of the most eye-catching cultural scenes in the new century. Especially in recent years, with the development of new media technology and the popularization of mobile digitalization, network literature and art have ushered in a broader space for development [1]. Not only has the number exploded, but it has also achieved fission-type communication through multichannel communication, multiplatform display, and multiterminal push. It not only enriches the spiritual and cultural life of the people but also faces severe challenges to its quality.

In 2014, General Secretary Xi Jinping pointed out at the Symposium on Literature and Art Work that Internet technology and new media have changed the form of literature and art. It gave birth to a large number of new types of literature and art and also brought profound changes in the concept of literature and art and the practice of literature and art [2, 3]. Due to the development of digitization of characters, imageization of books, and online reading, literature, art and even social culture are facing major changes. It is necessary to adapt to the development of the situation, do a good job in the production of online literature and art creation, and strengthen the positive guidance.

In order to do a good job in the construction of online literature and art, the Central Committee of the Communist Party of China issued the *Opinions on the Prosperity and Development of Socialist Literature and Art* in October 2015, which for the first time clearly proposed to vigorously develop online literature and art. General Secretary Xi Jinping pointed out that “Cyberspace is the common spiritual home of hundreds of millions of people. Cyberspace is in line with the people's interests with clear sky and good ecology. Cyberspace is smoky and ecologically deteriorating, which is not in line with the interests of the people.” In order to give full play to the leading role of socialist ideology, it is necessary to strengthen the active and correct guidance of network literature and art. Not only is it of great significance to purify cyberspace and make online literature and art better benefit the people, but it is also a new topic for building a socialist ideological discourse system in the new era [4–6].

In 2018, at the National Propaganda and Ideological Work Conference, General Secretary Xi Jinping further emphasized that “the improvement of quality should be the lifeline of literary and artistic works, and more healthy and high-quality online literary and artistic works should be launched.” As a new thing, online literature and art has been highly valued by the party and the state in recent years and has increasingly become the research focus of the academic circles [7].

Therefore, actively research and judge the new changes, new characteristics and new trends of online literature and art in the new media field, accurately control the communication characteristics and laws of online literature and art, and actively and effectively regulate and guide it. It is of great significance for expanding and deepening the theoretical research of network literature and art, cultivating a good network literature and art ecology, and promoting the healthy development of network literature and art.

## 2. Overview and Development Trend of Network Literature and Art

### 2.1. Overview of Network Literature and Art

At present, there are still big differences in theoretical understanding and evaluation of network literature and art. There is still no clear consensus on its conceptual analysis. Therefore, it is necessary to cut into the two categories of “network” and “literature and art,” respectively, and carry out an ontological interpretation of network literature and art from the aspects of connotation, extension, and characteristics.

“Network” refers to the use of modern computer technology and physical electronic pulse technology. Through the mutual conversion between digital signals and electronic pulses, a virtual platform for information transmission, reception, and sharing is achieved. Using the network can connect any information terminal equipment that is openly associated with it to realize the sharing of information and resources among points, lines, surfaces, and bodies. With the introduction of electronic products such as computers, smartphones, and tablet computers into thousands of households, people can easily read words with the help of the Internet, and it is becoming more and more difficult to separate them.

The concept of “literature and art” is still controversial in the academic circles. One view holds that literature and art are collectively referred to as literature and art. Another point of view is that literature and art refer to literature, which is a parallel relationship with art [8]. In 2011, in the reform of the division of my country's discipline system, art, which originally belonged to the category of literature, was listed separately and became the thirteenth discipline category. This ended the history of subordination of art to literature in the division of disciplines for more than one hundred years. Combined with the current public context, it is clear that the former view is more reasonable and practical. That is, literature and art include various art forms such as literature and drama, music, dance, art, calligraphy, photography, folk art, acrobatics, film, and television.

As a new style of literature and art, “Internet literature and art” refers to the collective name of various literature and art forms that are published and disseminated through network platforms after informatization processing. In terms of its extension, it not only covers new art forms created by netizens such as online animation, online performances, online dramas, micromovies, online music, talk shows, and jokes. It also includes networked works of traditional literature and art such as literature and drama, music, dance, art, calligraphy, photography, folk art, acrobatics, and film and television. Compared with traditional literature and art, network literature and art mainly have the following four characteristics:

1. The main body of creation is based on the mass netizens. Although there are some traditional literary and artistic workers in the main body of online literature and art, the main source is still ordinary netizens with “grassroots.” They come from different social classes, with different occupational backgrounds, and the number of groups is huge.
2. The content of the works is expressed as “more than good.” Compared with the orthodoxy of traditional literature and art, online literature and art tend to be more entertaining. Although there are many excellent works, under the influence of consumerism and market economy, the production of online literature and art is inevitably mixed with some vulgar and vulgar content, resulting in uneven quality of their works.
3. The means of communication is digital media. Only when complex information such as words, pictures, images, and data in online literary and artistic works are transformed into digital models, and then into computer binary codes, can the dissemination process of works on the Internet be completed. This is the most essential difference between network literature and traditional literature and art.
4. The audience is mainly the younger generation. Compared with traditional literature and art, which is “suitable for all ages,” the audience of online literature and art is mainly concentrated in the young generation of “post-80s” and “post-90s.” Among them, the number of readers of online literature alone is as high as more than 200 million, and most of them are young people. This makes online literature and art closely related to the daily life of young people, has a wide impact on their thoughts and behaviors, and is manifested as a “fan” culture.

### 2.2. The Development Trend of Network Literature and Art

Network literature and art is a new type of art form that is generated and developed relying on network technology. As far as its “connotation” is concerned, “Internet literature and art is endowed with Internet artistic thinking under the influence and influence of Internet technology, new media, and social changes. It represents the life of the times and expresses modern experience and thoughts and feelings with new artistic production methods. In essence, it is mainly reflected in three aspects: Internet artistic thinking, new art production methods, and aesthetic art.

From the perspective of the development of online literature and art, it mainly includes text-based online novels, online poems, video-based online dramas, online variety shows, online movies, online animations, online games, online performances, audio-based online music, and mobile phone value-added. In terms of development trend, it is mainly characterized by scale and industrialization, technologicalization and mobilization, and the integration and innovation of network literature and art and traditional literature and art.

#### 2.2.1. The Scale and Industrialization of the Development of Network Literature and Art

Data show that as of March 2020, the number of netizens in my country has reached 904 million, and the Internet penetration rate has reached 64.5%. Among them, the number of mobile Internet users reached 897 million, and the proportion of Internet users using mobile phones to access the Internet reached 99.3%. The proportion of using TV to surf the Internet was 32.0%. The proportions of using desktop computers, laptop computers and tablet computers to access the Internet were 42.7%, 35.1% and 29.0%, respectively [9].

In terms of user scale and utilization rate, online literature and art have shown a dual trend of huge numbers and further growth. As of March 2020, the scale of online music users was nearly 635 million, accounting for 70.3% of the total netizens, and the scale of mobile phone users was nearly 633 million, accounting for 70.5% of mobile netizens. The scale of online literature users reached 455 million, accounting for 50.4% of the total netizens, and the scale of mobile phone users reached 453 million, accounting for 50.5% of the mobile netizens. The scale of online game users is nearly 532 million, accounting for 58.9% of the total netizens, and the scale of mobile phone users is nearly 529 million, accounting for 59.0%. The number of online video users reached 850 million, accounting for 94.1% of the total netizens, of which the number of short video users was 773 million, accounting for 85.6% of the total netizens. These data show that the huge number of users, diverse forms of expression, continuous growth scale, and positive development trends have created the basic style of online literature and art.

From the perspective of industrial development, network literature and art not only enrich the social and cultural life of the public but also become an important part of the cultural industry and network economy in the new era.

At present, the network literature and art industry has many subdivisions, forming the basic pattern of “one superpower, many strong.” Data in 2019 show that online games have occupied “half of the country” in the online literature and art industry in terms of total volume, and its total output value of 133.96 billion yuan accounts for half of the entire industry scale. Online live streaming ranked second, reaching a scale of 64.92 billion yuan, which has surpassed the market size of Chinese cinema movies (60.98 billion yuan, 2018). The industries that have reached a scale of 10 billion yuan include online literature (15.73 billion yuan), online dramas (12 billion yuan), online animation (15 billion yuan), and short videos (14.01 billion yuan). The industrial scale of other online literature and art segments, including online variety shows (6.7 billion yuan), online movies (3 billion yuan), online music (6.26 billion yuan), and online audio (4 billion yuan), has also reached dozens billion scale.

It can be said that many subfields have achieved large-scale and industrialized development. It should be noted that due to the “savage growth” of Internet literature and art [10]. As a result, its industrial development is not mature enough, and its industrial attributes are not clear enough. Investment and financing, industrial chain, and profit models all need to be explored urgently.

#### 2.2.2. Technicalization and Mobility of the Development of Network Literature and Art

The overall promotion of digitization and networking is complementary to the personalized diversification of the emerging online literature and art market. This is of great significance for improving the supply capacity of network cultural products and services and improving the quality of cultural services. At the same time, it also promotes the healthy development of network literature and art.

Benjamin believes that “every form of art has gone through a critical stage in its development history, and it can only be effective under the change of new technologies. In other words, it needs to rely on new forms of art to require breakthroughs.” The advancement of technology promotes with the evolution of network art form and the development and change of art style. In the development of Internet literature and art, the trend of integration of Internet technology and art has become increasingly prominent. It promotes the continuous dissolution of the boundary between art and technology and affects people's artistic aesthetics and technology through the media and wider means and channels of the Internet.

Online literature, online games, online movies, online short videos, and online animation are all based on new network technologies. Combined with the integration of artificial intelligence and other aspects across technical levels, rich works of art have been created. And in the blending of modern media and multiculturalism, a new artistic concept is constructed. For example, the use of special effects in online movies can bring the ultimate visual pleasure to the audience, and virtual reality (VR) technology has broken through the traditional art aesthetic method of “contemplation.” By creating an immersive multidimensional dynamic sensory world, it extends the audience's senses and brings an “immersive” aesthetic experience to the audience.

With the popularization and wide application of smart large-screen mobile phones, the user scale and penetration rate of mobile network video, online music, online games, and online literature continue to grow [11]. The mobile characteristics of network literature and art dissemination-acceptance are gradually obvious. The mobilization of dissemination-acceptance not only profoundly affects the creation and production of online literature and art but also the habits and stereotypes of people's aesthetic acceptance. It also inspired and spawned new forms of artistic expression, such as the rise of vertical screen dramas. Based on the portability of mobile devices, it is also compatible with the fast-paced lifestyle of users and the characteristics of receiving high-density and fragmented information anytime, anywhere. Mobility makes many online literary and artistic works present the characteristics of single content and short episodes.

#### 2.2.3. Fusion and Innovation of Internet and Traditional Literature and Art

In recent years, the development forms of online literature and art have become increasingly rich, and at the same time, the integration and innovation with traditional forms of literature and art has also been deepened. Its remarkable performance is that with the improvement of quality, the distinction and boundary between online literary and artistic works and traditional literary and artistic works are increasingly blurred. Especially in the field of online audio-visual, excellent online variety shows, online dramas, and online movies are difficult to completely distinguish from TV variety shows, TV series, and cinema movies. Not only that the play mode of “from network to station” program interpenetration and location transfer further makes up for the differences and boundaries between the two.

Looking at the production of online literature and art in recent years, on the one hand, mobile Internet communication with mobile phones as the main carrier occupies a dominant position. New forms of communication such as WeChat, Weibo, Weibo, Weibo, Internet TV, and digital newspapers and periodicals have become the main channels for the public to obtain information and relax and entertain.

Network literature and art have different characteristics and laws from traditional literature and art because of the evolution of language and thinking. With its distinctive personality and innovative power, it has changed the pattern and trend of traditional literary and artistic creation and production and has increasingly radiated, driven, and even led in enriching practice. On the other hand, the advantages of historical resources and development experience of traditional literature and art cannot be ignored. The interaction, mutual influence, and mutual cooperation between online literature and art and traditional literature and art have become an important trend of media integration and have also profoundly changed the pattern of media and literature and art.

Therefore, in the in-depth transformation of “Internet + literature and art,” on the one hand, the characteristics and advantages of traditional literature and art are further exerted, and at the same time, it is also reversed to learn from and absorb the new experience of network literature and art. On the other hand, in terms of development trends, if we say that the “transformation” of online literature and art has already begun, the “change” of traditional literature and art has been latently growing. Then, the fusion and innovation of the two is essentially the transition of aesthetic discourse from transition to transfer in the intersection of “tradition and modernity.” And make the new laws of literature and art precipitate and condense in the field of literature and art, and then move towards the process of “new normal” and “new common name.”

## 3. Communication Characteristics of Network Literature and Art

Under the background of the Internet, the network literature and art communication show remarkable characteristics such as the entertainment of the communication target, the diversification of the communication subject, the younger of the communication audience, the flattening of the communication content, and the digitization of the communication form.

### 3.1. Entertainment of Communication Target

As we all know, the practice and exploration of online literature and art are carried out in the context of the prevalence of consumerism culture. From the perspective of the dissemination goal of online literature and art, the creators of online literature and art initially created with an entertainment attitude to meet the public's pleasure needs.

In the context of the consumer society, the theme of art in online literature and art has become relaxed and casual. Art no longer undertakes serious missions of enlightenment, encouragement, and criticism, but like a string of beautiful and ugly bubbles appearing rapidly, but broken again in an instant. This is an era of loud noises. Although the spirit of enlightenment, encouragement and criticism is no longer serious, the expression of ideas through works of art is still popular. It is just that this expression often takes on a strong, uncondensed emotional tone.

Therefore, to satisfy people's leisure and relaxation spirit as the main purpose, to entertain themselves and share entertainment as the goal, and to promote and realize the flow of capital logic for the purpose of consumerism is wrapped in it. Behind this consumerist approach is the advent of the era of national entertainment, and the cultural concepts of “entertainment until death” and “happy is good” are rampant. People's pursuit of daily spiritual life and the improvement of spiritual quality make online literature and art meet people's inner needs. As a result, it becomes people's way of life, way of life and communication, and shapes the world in which people live. Changes and even subverts the experience history, thinking logic and aesthetic concepts handed down in people's daily life and traditional society.

With the prosperity of consumerism and entertainmentism, the development of online literature and art gradually tends to be “fashionable, commercialized, and profitable.” The phenomenon of “demoralization, dehistoricalization, and devaluation” in the process of online literature and art dissemination has attracted people's attention.

### 3.2. Diversification of Communication Subjects

At present, the main body of online literature and art communication consists of four types: UGC (User Generated Content), PGC (Professionally Generated Content), PUGC (Professional User Generated Content), and OGC (Occupationally-generated Content). UGC is the most common dissemination subject. Weibo, live broadcast, Douban, and forums can all be regarded as UGC.

With the opening of various network platforms to users, users upload and share content, which further promotes the development of UGC. PGC is a communication subject that is developing rapidly at present. For example, Youku, Tencent, iQiyi, and Himalaya all focus on professional content production. Through a professional content production team, a unified standard and normative form can be established, so as to ensure the quality of the content and satisfy the user's good experience. PUGC is a new model which is a fusion of UGC and PGC. Generally, it is a platform organization such as a studio or company that produces professional content. Well-known celebrities in the industry generally adopt this model, such as Gao Xiaosong's *Xiao Shuo* and Wu Xiaobo's *Wu Xiaobo Channel*.

OGC is based on some specific content such as news hotspots, financial comments, artistic aesthetics, and works appreciation. This is a form of content production created by a group of experts to meet the needs of a specific group. From the development history of major video websites, we can see that their communication subjects are increasingly diversified.

Taking Bilibili as an example, the early Bilibili was mainly based on user-uploaded videos, which contained a lot of UGC content. For example, secondary creations such as mixed cutting of original works, and with the transformation of the website ecology, a large number of professional institutions have settled in Bilibili, and PGC content is increasing day by day. In recent years, Bilibili has grown into a website with a high viscosity community culture and user increment with the help of PUGC content. In addition, NetEase Cloud Music integrates UGC, PGC, and PUGC modes. On its APP, there are not only the works of independent singer-songwriters but also the singings of singers from major music companies, as well as songs by fans and other music enthusiasts.

These all indicate that the main body of communication of network literature and art presents the characteristics of diversification. Inject new vitality into the production and development of online literature and art. It also brings many problems such as plagiarism of works, the proliferation of piracy and the protection of literary and artistic copyrights and rights protection, which need attention and effective management.

### 3.3. Youth of Communication Audience

Data show that as of March 2020, my country's netizens are still dominated by young people. The 20- to 39-year-old group accounted for 52.3% of the total netizens, and the 20 to 29-year-old group accounted for the highest proportion, reaching 21.5%. Young people are the main audience of online literature and art. Therefore, the content, subject matter, form of expression, language structure, ideological concept, and spiritual expression of online literary and artistic works all need to grasp the psychology of young audiences and are more in line with the tastes and needs of young people and online generations [12]. At the same time, young audiences have long been immersed in Internet culture. It is well versed in various Internet hotspots and emerging vocabulary and is familiar with “stalks” with unique meanings on the Internet. Therefore, online literature and art has become a unique field for them to communicate and identify.

Different online literature and art communication platforms have different audience groups. The core users of Bilibili are two-dimensional animation enthusiasts and radiate the majority of young people. Douban's audience is mainly literary youth. Kuaishou and Douyin also have fixed audiences. These users show the characteristics of “net generation,” the virtual cyberspace is their common memory of growth, and the social attributes between users also show a certain virtuality.

Bilili's partitions show differences in their communities, and each individual user may have attributes of different communities at the same time. Fan opera area, game area, entertainment area, and film and television area have gathered a large number of fans. They communicate and communicate through various methods such as “barrage” and text comments, showing a certain degree of sociality. The fans of each community have a certain amount of expertise in the community's field, as well as a deep understanding of the subcultural terminology and social principles of their group.

From this perspective, the audience of online literature and art is increasingly showing the characteristics of community and circle. These characteristics, in turn, guide the main body of online literature and art to fully consider the desires, interests, and preferences of the audience, especially young people, when carrying out literature and art production and dissemination [13]. It may make the production and dissemination of online literature and art focus on “market orientation” and “consumption orientation,” while ignoring “cultural orientation” and “education orientation.” It has a negative impact on the healthy development of young people's world outlook, outlook on life and values.

### 3.4. Planarization of Communication Content

Online literature and art in the form of online music, online TV, online movies, online games, and online short videos enable interpersonal “communication” to easily transcend the walls of time, space, and even power and class and achieve “everyone to everyone.” In terms of dissemination content, it basically shows the characteristics of flat, perceptual, and daily life. In recent years, “short videos” such as Douyin, Kuaishou, and Volcano have sprung up as short video programs or “miniaturized” light variety shows. The short video is 15 seconds to 3 minutes in length, short and concise, fast-paced, strong in social networking, and highly topical. Coupled with the vertical subdivision of themes, it is deeply welcomed by young users and respected by major platforms.

This “simple and fast” communication method also meets the needs of people's daily entertainment. The dissemination content presents the characteristics of flat and intuitive, classified presentation, massive time-sharing, personalized customization, precise orientation, and unlimited links to similar works. In essence, it reflects the characteristics of daily life narrative, realistic narrative, individualized narrative, and liberalized narrative. This dissemination of content that focuses on flat, perceptual, real-time, and life-like content makes people gradually adapt and get used to replacing text reading by electronic reading pictures. Sound, color, light, and shadow replace understanding and imagination, and visual pleasure melts rational thinking, resulting in the phenomenon of subject dissolution or sinking [3, 14].

### 3.5. Digitalization of Communication Form

Since the new era, online literature and art have paid more attention to the three-dimensional effect, emphasizing emotional rendering and atmosphere creation, striving to achieve a whole-hearted immersive experience, and do their best to provide audio-visual entertainment. Especially driven by digital imaging technology, network hypertext technology, and multimedia technology, the production of network literature and art increasingly relies on digital “simulacrum.” Digitization, audio-visualization, simulacra, and intellectualization have become the dominant trends in contemporary online literature and art dissemination. Digital new technologies such as virtual reality (VR), augmented reality (AR), and cloud gaming platforms are gradually entering the homes of ordinary people. Their large-scale popularization has played a role in promoting the dissemination of literary and artistic works.

The application of new technologies such as artificial intelligence, big data, cloud computing, and blockchain has greatly freed the communication of literature and art from the constraints of time and space. To further enrich personal aesthetic experience, the forms of online literature and art communication are also more diverse. The popularization of 5G networks in the future will bring the speed of information dissemination to a new level. Its application will expand the breadth and depth of network communication channels and make online communication of high quality, high-quality audiovisual works a reality. It also enables the realization of a cross-time, cross-regional art appreciation mode, and you can use 5G networks and VR equipment to visit art galleries and museums at home [15].

The large-scale application of new technologies, new equipment and new media will diversify the forms of online literature and art dissemination. The rich communication channels will also continuously improve the viewing experience of users and meet the needs of different types of cultural consumption.

It should be noted that the digital production and dissemination of online literature and art has also made contemporary spiritual culture sharply inclined to focus on feelings, desires, and bodies. Replacing humanistic connotation and aesthetic inner discipline with technicalism is likely to lead to the disappearance of literary and artistic nature. The proliferation of virtual images and the origin of information worship will lead to the degradation of aesthetic experience and the passivation of aesthetic rationality. As a result, the liberating power of technology has been alienated into the shackles of the development of network literature and art.

## 4. Guiding Strategies of Network Literature and Art

Through the current creation and dissemination of new experiences, new features, and new trends, we can see the rapid development of network literature and art. On the one hand, the rapid development of online literature and art shows the great power and vitality of “Internet +.” At the same time, it also has a profound impact on people's daily life, aesthetic taste, cultural psychology, values, as well as the fashion of the times, ideology, and social development [7, 16]. On the other hand, there are also various problems behind the development of online literature and art such as entertainment, vulgarity, and vulgarity in the production of online literature and art emerge in an endless stream.

The problem of copyright protection of online literature and art is prominent, and the fast-food, flat, and superficialization of online literature and art consumption has gradually become a trend. The economic and social benefits of Internet literature and art dissemination are separated from each other, the technologicalization of Internet literature and art development has eliminated the human nature of literature and art, and so on. All these require us to face up to the cultural guidance and management norms of network literature and art, improve the network literature and art governance system, purify the network literature and art ecology, and promote the healthy development of network literature and art.

### 4.1. Promoting Integrity and Innovation

“Keeping the righteousness” is the basis for the creation and production of online literature and art. This includes two main aspects: adhering to the development direction of socialist literature and art with Chinese characteristics and following the laws of network literature and art development. From the perspective of the former, socialism with Chinese characteristics is the institutional soil for the survival of the majority of the people. The socialist core values are closely related to the people's living conditions and spiritual aspirations. It reflects the basic moral ideals and value orientations that people should uphold when integrating into social life.

Adhering to the development direction of socialist literature and art with Chinese characteristics requires that online literature and art must strictly distinguish the boundaries between popular and vulgar, vulgar, and vulgar, and online literature and art should not become synonymous with “three vulgar” cultures [17]. It cannot become a gathering place for distorted mentality, extreme emotions, and abnormal psychology. Socialist core values are still the basic background of online literature and art. As far as the latter is concerned, as a new type of literature and art format, online literature and art has its own vitality, uniqueness of media and communication. Only by earnestly following the particularity and dissemination law of network literature and art's own development. In order to make the best use of the situation, promote the innovation of online literature and art.

“Innovation” is based on a firm and correct political orientation and value orientation. Actively promote the innovation of the concept, content, and form of online literature and art, so that the production of online literature and art can closely follow the pulse of the times, be close to real life, and reflect the spirit of the times. Face up to the entertainment, flat, diversified, youthful, digital, and other characteristics of online literature and art communication. Give full play to the features and advantages of new media in terms of interactivity, mobility, and immediacy. Innovate the theme discovery, narrative paradigm and artistic skills of online literature and art, and develop and innovate in related fields such as technology, industry, and communication.

Pay special attention to the large number of young audiences, and carry out artistic innovation according to their youthful, socialized and personalized characteristics. Create a youth culture in the new era and make young people the pioneers of the progress of the times. Teenagers are not only the inheritors of China's excellent traditional culture but also the ones responsible for the great rejuvenation of the Chinese nation.

### 4.2. Create a Good Network Literature and Art Ecology

The report of the 19th National Congress of the Communist Party of China pointed out that it is necessary to “strengthen the construction of Internet content, establish a comprehensive network governance system, and create a clear and clear cyberspace.” In recent years, in response to many chaos and problems in the field of online literature and art, relevant departments have promoted the application of traditional laws to the Internet and established special legislation in the Internet field. A multilayer law-based Internet governance system has been established, with the *Administrative Measures for Internet Information Services* as the basic regulations and special management measures for online audio-visual, online publishing, online literature, online live broadcast, and online games as the main content.

Laws such as the Cybersecurity Law, the Film Industry Promotion Law, and the Criminal Law Amendment (IX) have been passed, and the Measures for the Administration of the Internet and Other Information Network Dissemination of Audio-Visual Programs, the Regulations on the Administration of Internet Audio-Visual Program Services, and the Internet Provisions on the Administration of Publishing Services, “Interim Measures for the Administration of Internet Advertisements,” “Regulations on the Administration of Internet Live Streaming Services,” “Notice on Strengthening the Copyright Management of Online Literary Works,” “Regulations on the Administration of Internet Forum Community Services.” It provides an institutional guarantee for correcting the ecological imbalance and chaos of online literature and art, creating a clean and positive cyberspace, and promoting the healthy development of online literature and art.

In 2016, the State Administration of Press, Publication, Radio, Film and Television issued the *Notice on Further Strengthening the Planning and Management of Original Audio-Visual Programs on the Internet*. In response to the problems of too many film and television stars, star chasing, pan-entertainment, high-priced film remuneration, and fraud in ratings (click-through rate) in some literary and artistic programs, it is emphasized that we must firmly grasp the correct political direction and strengthen value guidance. Adhere to the people-centered creative orientation and resolutely curb bad tendencies such as star chasing and star speculation and pan-entertainment. Encourage high-quality content to win, constantly innovate program forms, and strictly control the remuneration of guests. Strengthen the governance of TV dramas and online dramas (including online movies) to promote the sound development of the industry. Strengthen the use and management of ratings (click-through rate) survey data, and resolutely crack down on the fraudulent behavior of ratings (click-through rate).

In 2017, the State Administration of Press, Publication, Radio, Film and Television issued the *Notice on Further Strengthening the Management of the Creation and Broadcasting of Online Audio-Visual Programs*, putting forward further requirements for the creation and broadcasting of online audio-visual programs. The notice pointed out that all kinds of online audio-visual programs must adhere to the aesthetic bottom line of civilization and health. Entertainment reports must respect morality and art and must not use the hype of scandals and privacy scandals as gimmicks to gain click-through rates.

Online variety shows, online dramas, and online movies must resolutely oppose unhealthy trends such as sky-high star chasing, boring games, and luxurious feasts and avoid promoting the game life mentality and exaggeration [18]. In addition, in view of the outstanding problems existing in the online video industry, online live broadcast and short video websites have been urged to self-check and correct themselves. Promote Internet companies to enhance their sense of responsibility and strengthen management measures. The Ministry of Culture and Tourism has organized online performances, centralized law enforcement inspections in the online game market, cleaned up prohibited content in the online cultural market, and standardized the order of elites in the online cultural market.

It is worth noting that for network platforms and operators, supervision measures still need to be further improved. For example, user identity verification is enabled for short video platforms, and content is selectively displayed to minors. The online platform is obliged to review and deal with online works and punish those works that are shoddy for rubbing hot spots and IP, works with vulgar and vulgar content, and works that spread obscenity, pornography, bloody violence. Effectively restrict minors' access to online games to prevent teenagers from indulging in online games.

### 4.3. Establish the Awareness of Network Literature and Art

In March 2019, General Secretary Xi Jinping pointed out: “A country and a nation cannot be without a soul. Culture, literature and art, philosophy and social sciences belong to Bacon's soul-building work, occupying a very important position in the overall work of the party and the country, and insist on and develop Chinese characteristics in the new era. It plays a very important role in socialism.” In the era of all media, establishing the awareness of “quality is king” and promoting the quality of online literature and art production is the only way for the development, transformation and upgrading of online literature and art, and it is also the meaning of the title of realizing the function of “bacon casting the soul” of online literature and art.

The connotation of “high-quality products” of online literature and art includes two levels. One is the boutique in the sense of “product.” At the “product” level, quality means the intensive cultivation of online literature and art in terms of production, dissemination, and service. For example, in terms of production, the industrialized production process of online literature and art has become increasingly clear, the division of labor has become increasingly refined, and the application of technical means has become increasingly mature. This is the basic guarantee for the production of high-quality products. In terms of dissemination and service, accurate dissemination of literary and artistic works, finding suitable audiences, meeting the spiritual needs of audiences, and providing good postservice services are all elements and awareness of online literary and artistic works. The second is the fine product in the sense of “work.” At the level of “work,” quality means the improvement of online literature and art in terms of content and value.

High-quality content is the decisive factor for the sustainable development of the online literature and art industry. Therefore, online literature and art should reflect the life of the times, demonstrate the spirit of the times, take truth, and tell Chinese stories. As emphasized in the report of the 19th National Congress of the Communist Party of China, “to prosper literary and artistic creation, adhere to the unity of profound thinking, exquisite art, and excellent production, strengthen the creation of realistic themes, and constantly launch masterpieces that praise the party, the motherland, the people, and the heroes.

In terms of value goals, the development of online literature and art should take “Bacon casts the soul” as its value appeal. Consolidate hundreds of millions of netizens with Xi Jinping Thought on Socialism with Chinese Characteristics for a New Era and actively cultivate and practice socialist core values.

In terms of formal requirements, online literature and art must not only be “down-to-earth” but also “popular.” “Grounding Qi” means to truly express the feelings, thoughts, hopes, and wishes of the people living on our land. “Gathering popularity” means that the form is popular, and it should warm people, infect people, educate people, unite people, inspire people, carry forward the truth, goodness and beauty, and transmit positive energy.

## 5. Conclusion

In the context of the continuous development of digital, intelligent and networked emerging technologies, it has had a profound impact on the creation and dissemination of online literature and art. But at the same time, we should keep in mind that culture is the foundation of the lasting innovation and development of network literature and art. Network literature and art should grasp the laws of digital and new media communication development and build a comprehensive and three-dimensional Chinese-style strategic communication system. In order to meet the spiritual and cultural needs of the people and the mission of spreading Chinese culture to the outside world, we will continue to create high-quality, high-standard masterpieces that can stand the test of the international market and the test of people around the world.

## Data Availability

The dataset can be obtained from the author upon request.
